# Research on Classroom Online Teaching Model of “Learning” Wisdom Music on Wireless Network under the Background of Artificial Intelligence

This article has been retracted.

**DOI:** 10.1155/2021/3141661

**Published:** 2021-11-27

**Authors:** Jie Shan, Muhammad Talha

**Affiliations:** ^1^Music Department of Tangshan Normal University, Tang Shan, He Bei 063000, China; ^2^Department of Computer Science, Superior University Lahore, Pakistan

## Abstract

This article uses a multimodal smart music online teaching method combined with artificial intelligence to address the problem of smart music online teaching and to compensate for the shortcomings of the single modal classification method that only uses audio features for smart music online teaching. The selection of music intelligence models and classification models, as well as the analysis and processing of music characteristics, is the subjects of this article. It mainly studies how to use lyrics and how to combine audio and lyrics to intelligently classify music and teach multimodal and monomodal smart music online. In the online teaching of smart music based on lyrics, on the basis of the traditional wireless network node feature selection method, three parameters of frequency, concentration, and dispersion are introduced to adjust the statistical value of wireless network nodes, and an improved wireless network is proposed. After feature selection, the TFIDF method is used to calculate the weights, and then artificial intelligence is used to perform secondary dimensionality reduction on the lyrics. Experimental data shows that in the process of intelligently classifying lyrics, the accuracy of the traditional wireless network node feature selection method is 58.20%, and the accuracy of the improved wireless network node feature selection method is 67.21%, combined with artificial intelligence and improved wireless, the accuracy of the network node feature selection method is 69.68%. It can be seen that the third method has higher accuracy and lower dimensionality. In the online teaching of multimodal smart music based on audio and lyrics, this article improves the traditional fusion method for the problem of multimodal fusion and compares various fusion methods through experiments. The experimental results show that the improved classification effect of the fusion method is the best, reaching 84.43%, which verifies the feasibility and effectiveness of the method.

## 1. Introduction

The integration of artificial intelligence and education has triggered a change in the concept of music teaching in colleges and universities, the restructuring of the relationship between teachers and students, and the change of learning methods. Facing the opportunities and challenges brought by artificial intelligence technology, it is necessary to think about the value of artificial intelligence technology to the music teaching scene and method reform in colleges and universities, the integration of subject horizons, and the improvement of sight singing is given [1]. It is necessary to continuously explore the path of reforming music teaching in colleges and universities by building databases and intelligent sampling and deeply consider the feasibility and boundaries of music teaching reform in colleges and universities from the perspectives of music theory, educational laws, and technological progress [2]. Due to the emergence of computer technology, intelligent sequence software related to it continues to be available on the market. Computers begin to interact with synthesisers and music workstations as a central system to create MIDI (Musical Instrument Digital Interface) digital music system, a more intelligent music operating system. [3]. When the digital music system is used in music classroom teaching, it means that the teacher's teaching has a powerful teaching aid system, and it also means that the learning of music knowledge and the practice of music skills have taken place [4].

Knowledge acquisition has never been more democratic or convenient than it is today, thanks to the digital era. Knowledge may be tested everywhere and at any time under specific technological circumstances [5]. Education started to stress internalisation and development of individual knowledge when the acquisition of indirect human experience became convenient [6]. Students' experiences should be a major focus in music education. Students may quickly acquire musical symbols and music expertise by using digital music platforms. Resegmenting time and removing space restrictions are required. Teachers must reexamine the goal, methodology, structure, and assessment techniques of teaching. Since the MIDI data two-way switch has been developed successfully, wireless networked instruction in music schools has become a reality. They may freely share MIDI information with one another. The intelligent tutoring system (ITS) was created in the early phases of the application of artificial intelligence in education, and it is the most popular technique of integrating artificial intelligence with education as well as the future growth direction of the teaching system [7–9]. As a result of this evaluation and processing, the intelligent teaching system may choose learning materials that are suitable for students' levels and interests as well as conduct ongoing analyses and give students with feedback on their classroom performance. The development of the intelligent teaching auxiliary training system is to apply artificial intelligence technology to the test training link in the teaching link, and the complete examination process undertaken by the teacher in the past is handed over to the computer system to complete, not only can the teacher be relieved from the heavy work, the burden is liberated, and the high efficiency and high accuracy of the test process can also be improved. The effect of combining music itself and lyrics to intelligently classify music is to a certain extent better than that of single-modal intelligent classification based on audio features or lyrics features. Therefore, this article studies multimodal intelligent music online teaching. While performing intelligent classification, use lyrics to intelligently improve classification accuracy, categorise music, and mix the two using a fusion technique. To begin, the lyrics are represented using the vector space model (VSM) in artificial intelligence processing technology, which adds word frequency information and document frequency information as the weight of features. Second, an enhanced wireless network node feature selection technique is presented and compared to the conventional wireless network node feature selection method while choosing lyrical features. Then, we use latent semantic analysis (LSA) to perform secondary dimensionality reduction on lyrics features to further remove redundancy. Finally, the wireless network model is used for classification.

## 2. Related Work

As a unique field in education, music education must follow the pace of informatization in order to develop. Mobile Internet has promoted the development of commerce, and the education industry uses wireless network technology in classroom teaching to enable students to learn and develop according to their own needs [10]. Big data, AI, and VR technologies have been changing the Internet education model. Building a professional online knowledge platform has become an urgent requirement of the times, and music education strives to build a social, teaching, feedback, learning, knowledge base, classification recommendation, etc. for comprehensive automated intelligent system.

Walton and Nayak [11] think that online education not only offers learning materials but also a tiny course with extra teaching content based on microresources from the viewpoint of learning. A full teaching framework, exercises, and curriculum are all included, as is an assessment of the learning effects. Microclasses, according to Cantu-Ortiz [12], are brief and succinct internet films that convey a specific piece of information and have learning or teaching purposes. Ideally, online courses should have a clear teaching objective and be no more than 10 minutes long. Talha [13] utilised a two-dimensional wisdom model to investigate the connection between music wisdom and five important characteristics of music signals (namely, melody, rhythm, loudness, spectral centroid, and texture). Since then, a large number of academics have stepped up their efforts and increased the depth and breadth of their study in this area. A music smart label prediction method based on a smart vector space model was presented by Talha et al. [14]. A more precise approach is to use a smart space vector model to extract wisdom words from the lyrics, then a support vector machine to gather music from the same genre as that to be categorised, and then apply a similarity calculation algorithm to perform all of the music in that genre.

At present, the most common method of smart music online teaching is audio-based smart music online teaching, that is, by extracting the underlying physical characteristics of music, analyzing and processing these characteristics, and then using machine learning methods to identify embedded music signals [15]. The underlying physical features include time domain features, frequency domain features, and cepstrum features of music. Short-term energy, short-term average amplitude, short-term average zero-crossing rate, short-term autocorrelation function, short-term average amplitude difference function, and so on are time domain features; frequency domain features are spectral centroid, spectrum roll-off, spectral rolloff point, spectral flux, and so on; cepstral features are mel frequency cepstral coefficient (MFCC) and perceptual linear prediction cepstral coefficient (PLPCC19). Şerban and Todericiu [16] proposed a new classification algorithm, the information unit mixing model (ICMM) to automatically classify music intelligence. ICMM is a three-tuple semantic structure based on fuzzy concepts and has obvious advantages in modeling high-dimensional concepts. In addition, ICMM is applicable to both unsupervised learning and supervised learning. Some scholars have proposed a music intelligence classification method based on a two-layer model. This method divides musical wisdom into four categories: angry, happy, sad, and peaceful. First, the calm class is used as the basic class, and then the support vector machine is used to train each target class and the base class, respectively, to obtain four wireless network models. Each test sample will get four predicted values, which are then used as the second, and the characteristics of the layered wireless network model are classified. It can be seen that the research on content-based smart music online teaching has achieved great results and is becoming more and more diversified [17].

## 3. Construction of an Online Teaching Model for Wireless Network Smart Music Classroom Based on Artificial Intelligence

### 3.1. Wireless Network Level Distribution

The main task of the musical wisdom cognitive model is to construct a classification function or classification model to map music from unknown wisdom categories to known wisdom categories. This model is also called a classifier, which predicts the category label of the music to be classified.  Figure 1 shows the hierarchical topology of the wireless network. The learning stage (or training stage, developing a classification model) and the classification step are the two major phases of smart music online education (using the model to predict the category of music to be tested).

In the first stage, the music in the training set is labeled in advance, and a classifier is constructed on this basis. The training set is composed of a music library and its corresponding category labels. This process is actually learning a mapping or function *y* = *f* (*x*), which can predict the class label *y* of a given ancestor *X*.

(1) $$\begin{array}{c} X\left[t\right]=\left\{t\in R\;|\;x\left(1\right),x\left(2\right),\cdots ,x\left(t\right)\right\}, \end{array}$$

(2) $$\begin{array}{c} y\left(n\right)=A*X\left(n\right)-t*x\left(n-1\right). \end{array}$$

In the second stage, the classification model is used to classify the given test set, the class label of each metagen to be tested is compared with the class prediction label of that metagen from the learning model, and the accuracy of the classification model on the test set is calculated. The fundamental concept is to compute the likelihood of each category occurring under the conditions under which the sample occurs, then choose the category with the highest conditional probability as the sample's category.

(3) $$\begin{array}{c} \bar{x^{2}}\left(t,n\right)-{\left|x\left(t,n\right)\right|}^{2}-2\left|\bar{x\left(t,n\right)}\right|*\cos\alpha =0, \end{array}$$

(4) $$\begin{array}{c} g\left(x,k\right)=\frac{1}{n}*\overset{n}{\underset{i=1}{\sum }}\left(1-\alpha \left(x\right)\right)\left(1-\beta \left(x\right)\right)*x\left(t\right). \end{array}$$

It is another classification algorithm widely used in data mining and machine learning, and its main purpose is to construct a knowledge structure that can guide the decision-making process. A decision tree is actually a tree structure, where each nonleaf node represents a test of a characteristic attribute, each branch represents a possible result of this characteristic attribute, and the leaf node represents a category.

(5) $$\begin{array}{c} \underset{i}{\sum }{\left|<\alpha \left(1\right),u\left(i\right)>\right|}^{2}+\underset{j}{\sum }{\left|<\alpha \left(2\right),u\left(j\right)>\right|}^{2}={\left\|u\left(i,j\right)\right\|}^{2}. \end{array}$$

The decision tree algorithm uses a top-down recursive method to determine the tree structure. It begins by testing the characteristics of the samples to be categorised one by one from the root node, then chooses its successor branches based on the tree structure, and ultimately arrives at the leaf node, where the category represented is the sample's category

(6) $$\begin{array}{c} \left\{\begin{array}{c} \phi \left(i,1\right)=\frac{\left(\phi^{+}\left(i\right)+\phi^{-}\left(i\right)\right)}{2},\\ \phi \left(i,2\right)=\frac{\left(\phi^{+}\left(i\right)-\phi^{-}\left(i\right)\right)}{2}. \end{array}\right. \end{array}$$

When this condition is established, the performance of the NBC method can reach the best. However, in reality, it is almost impossible for each feature to be completely independent and usually have a strong correlation, which greatly reduces the accuracy of the NBC method. Therefore, the NBC method is not more effective than other classification methods in practical applications.

### 3.2. Artificial Intelligence Algorithm Architecture

Online teaching uses microvideo as the core in a wireless network environment, supplemented by teaching design, forums, teaching courseware, learning guidance, exercises, tests, learning surveys, student evaluations, expert comments, teaching reflections, and question answers. The key factor of this model is the structure of the information processing system, which is composed of a large number of highly interconnected processing units, namely, neurons, which work in coordination with each other to solve problems together. ANN needs to be trained before pattern recognition or data classification to adjust the synaptic connections between neurons to adapt to the needs of different neural wireless network models. By categorising online teaching into parts and courses, the online learning platform efficiently manages a large amount of information. For online teaching, knowledge points and structure may be linked together and aggregated to create an acceptable and effective music knowledge system structure, which can offer various retrieval services such as categorization, topic keywords, or mind maps for online teaching. Factors influencing student engagement in interactive online courses are shown in Table 1. There are four main topics in this educational model: the teaching platform, the instructor, and the learning material, with the learner as the centre subject. The interaction between the four subjects creates the following interactive model.

For classification problems, the core idea of wireless networks is to find the optimal classification hyperplane to determine the decision boundary in the input space or high-dimensional feature space. The wireless network uses a set of labeled training data sets to construct a classification hyperplane (whether in the input space or high-dimensional feature space), which can separate positive and negative samples at the largest interval. In the case of nonlinearity, the wireless network uses the kernel function to map the input space to the high-dimensional feature space, transforming the nonlinear problem into a linear problem. Watching the video will clearly learn the content of the next day's class, which will greatly improve students' classroom communication and discussion capabilities. The purpose of data governance is to discover value. At the same time, high-quality data can also support the high value of data. Under the guidance of this idea, a value-oriented music curriculum data program is proposed, which includes 5 areas of activity: data integration and cleaning, continuous improvement of data quality, and data relationship combing, data mining and forecasting, and data visualization. Among these is the connection between data governance operations and other college and university business activities, in which the former provides the latter with a foundation for decision-making and business optimization, while the latter offers the former with a data source. Using the Internet infrastructure of “cloud + network + terminal,” focusing on teaching activities, student independent research, cooperative research, teaching resources, teaching materials, courseware, video, and animation design as means of teaching activities, using communication tools, face-to-face teaching video calls to set up a teaching environment with smart classrooms, and using big data.

### 3.3. Frequency Domain Analysis of Smart Music

The artificial intelligence teaching assistant system can realize two-way intelligent sampling for college music teaching and provide graphical analysis results. We take the sight singing and ear training course as an example, and two-way intelligent sampling includes selecting the content of the teaching materials and the content of the students. The intelligent sampling of the content of the teaching materials comes from the database, which contains all kinds of known music works, necessary materials for the sight-singing and ear training courses, and teachers' teaching methods. Music feature analysis is a very important step in the online teaching of smart music. Different music features may show different wisdom. Because of this, the primary goal of music feature analysis is to identify the optimal feature space for encoding musical information. As well as reflecting the wisdom of music, this feature area has to be unique enough to tell apart songs of varying wisdom. Using artificial intelligence's computation and self-thinking capabilities, these materials may be unified and integrated to provide the best answer for course teaching and assist instructors with preclass preparation. Students make up a large portion of the sample. In addition to the competition and sight-singing sections in the traditional content, it can provide a graph analysis based on the facial expressions, behaviour habits, receptive ability, and learning achievement matrix of the students, and finally let the teacher clarify the strengths and weaknesses of the students and intelligently analyse the appropriate training program and find specific training methods that are conducive to the development of students.

According to the design of the system, system users are divided into three groups: administrator, teacher, and student, and each group of users has different rights and refer to the functions of each user group, and design the functional structure of the system according to the composition of the system.  Figure 2 shows the line graph of the efficiency of the online system decision tree. Second, the decision tree is more efficient. It only needs to be constructed once, and then it can be used repeatedly, and the maximum number of calculations for each prediction does not exceed the depth of the decision tree. Decision trees, on the other hand, are more difficult to forecast for continuous fields, and they cannot make particularly precise judgements when dealing with huge data samples or many categorization categories. On the market, related intelligent sequence software is still accessible. Computers, synthesisers, and music workstations begin to operate together as a central system to create a more intelligent music operating system, known as the MIDI (Musical Instrument Digital Interface) digital music system. This music system is not only more comfortable for intelligent operation because of the computer connection but it also has improved information and data features.. Users can edit, modify, record, and play recorded MIDI messages at will. The elements are processed artificially. This high-tech teaching equipment has changed the traditional teaching methods, connecting teachers and students, and between students and students into a whole interactive relationship. It integrates traditional music symbols in a local area network in a digital and informatized manner. The scope of dissemination allows instant communication and exchange of information between teachers and students [18, 19].

### 3.4. Integration of Online Teaching Factors

For music teaching, the creation of scenes is conducive to the establishment of students' music learning psychology. The creation of the scene needs to be built on the basis of a large amount of data stacking and comparison. The artificial intelligence teaching aid system can collect and organize all kinds of sight singing and ear training content materials, including monophonic, interval, melody, and mode. Many additional music categories' contents are examined and compared once these fundamental ones have been collected and sorted, such as the comparison of piano timbre with tuba timbre under the same tune. The material you choose may appear in many instructional scenarios at any given moment. Sight singing and ear training are transformed into powerful tools for comprehending music as a result of this approach, which helps pupils learn faster and more efficiently. Advanced intelligent teaching methods have been adopted in higher music education for courses like composition, orchestration, and work analysis, which allows students to hear the notation and make changes in real time in their classrooms. The notation can also be used for various kinds of program editing and information processing.  Figure 3 depicts the system for integrating instructional factors on the internet.

The time domain characteristics of music refer to the time domain parameters of each frame calculated from the music signal. The design function of this management module is arrange the date of the examination, set the validity of the examination paper (examination papers that are not within the valid time range shall not be used or consulted), set the specific time for the release of the examination results of each subject, set whether to allow examinees to consult the test scores of related courses, set whether to allow candidates to view the standard answer sheets set for related test questions of the exams they are taking, and set whether to allow candidates to view the evaluation reports of the relevant course exams they have taken. Typical time-domain features include short-term energy, short-term average amplitude, short-term average zero-crossing rate, short-term autocorrelation function, and short-term average amplitude difference function are given. The short-term energy is a time series that allows us to track variations in the signal's energy over the course of a day. Generally speaking, voiced sounds have a higher short-term energy than unvoiced sounds, thus, the short-term energy sequence is able to tell the difference between the two with ease. As an added bonus, the beginning and finish points of music may be determined by looking at the short-term energy sequence instead. Most audio-based music characteristics are derived from voice signal properties. In the long run, speech signals' properties change, but the changes are gradual. Consequently, each frame is processed individually using the processing technique of stationary random signal and is split into consecutive small pieces. This is a technique for quickly processing voice signals. Time domain, frequency domain, and cepstrum are all types of audio characteristics.

## 4. Application and Analysis of Online Teaching Model of Wireless Network Smart Music Classroom Based on Artificial Intelligence

### 4.1. Artificial Intelligence Data Processing

The users of the system will put forward many specific requirements for the automatic test paper composition operation of the system according to the teaching task and the purpose of the investigation. The automatic test paper composition system must meet the requirements to the greatest extent. The specific content of each line is composed of various related control indicators of a specific test question in the question bank. These control indicators mainly include the number of the question, the type of the question, the chapter to which it belongs, and the difficulty of the question. It is represented in the system by binary code, with the particular content of each being the value of a certain index in the question bank. This article uses ASP. NET mobile control to realize the programming of mobile Web. We use Microsoft ASP. NET can quickly and efficiently design and write powerful Web applications for mobile devices. ASP. NET mobile controls are built in Microsoft. NET Framework, it will be Microsoft ASP. All the advantages of the .NET Web development model have been introduced into the field of mobile Web applications.

Since the calculation of short-term energy requires squaring, the difference between the magnitude and the amplitude is enlarged, and the characteristics of the short-term energy of the signal changing with time cannot be accurately reflected. As a result, a new feature called short-term average amplitude is suggested to describe the time-varying properties of signal energy. Short-term amplitude deviation data are shown in Figure 4 (below). If the adjacent sampled value exceeds the proper positive and negative threshold, it is evaluated whether or not to cross zero by distinct signs of adjacent sampled values. This means that crossing zero is not judged by adjacent sampled value signs. As a result, noise-induced erroneous zero crossings are eliminated. Unvoiced and noise often have a higher short-term average zero-crossing rate than voiced sounds, making it easy to tell the two apart using the short-term average zero-crossing rate. The short-term average zero-crossing rate, on the other hand, is an essential criterion for determining when music begins and ends. For every periodic signal, the short-term average amplitude difference function will be equal to the period's lag time or an integer multiple of the period.  Figure 5 depicts the music cycle signal's fan-shaped dispersion.

Experiments show that for frequencies below 1 KHz, the two have a linear relationship; for frequencies above 1 KHz, the two have a logarithmic relationship. MFCC is widely used in the field of speech recognition based on this connection. The voiced signal is approximately a periodic signal, so at a lag time point equal to the pitch period or an integer multiple of the pitch period, *k* will reach its minimum value. Using this property, we can distinguish between voiced and unvoiced sounds based on the *k* curve and estimate the pitch frequency of voiced sounds.

### 4.2. Realization of Online Teaching Model Simulation

Through the study of the operating rules of the examination system and the understanding of the teaching requirements of the course, the system adopts a semiautomatic test paper composition method. The instructor and the user write the subjective questions by hand, while the system intelligently composes the objective questions. The mathematical model applied to intelligent test paper composition is described. In the intelligent test paper composition system, the neural wireless network is introduced for further improvement. In order to verify the reliability of the system, a large number of simulation experiments were arranged. From more than 900 pieces of data collected in the experiment, about 600 sample data were selected for training, and the remaining more than 300 sample data were used for testing. It can be seen from the training effect that the BP algorithm has the problem of poor convergence. Even after 100,000 times of training, the convergence result is still not ideal, and there is still a certain gap from the set expected accuracy (0.01). It can be seen from the experimental results that the improved BP algorithm effectively solves the problem of poor convergence of the BP algorithm. After more than 1000 trainings, the convergence results are ideal and the desired accuracy is reached. (0.01), and the training speed is faster.

Figure 6 shows the vacancy rate curve of online teaching resources. According to the data dictionary during the demand analysis, we use the large-scale SQL Server 2000 database to design the database of the automatic answering system platform. The SQL Server 2000 database can basically meet the simultaneous access of small and medium-sized user groups. The database tables are designed according to the four major blocks of multimedia teaching system, student self-test system, personal document system, and teacher-student communication platform. System testing is the process of doing different assembly and confirmation tests using verified computer software and hardware, peripherals, wireless networks, and other components. The system test's goal is to see whether the multimedia information management system based on the mathematical campus fulfils the requirements specification's description. If not satisfied, we find out the discrepancies and propose a more appropriate solution. Audio performance test results: (1) when there are 29 people online, there is no delay in audio listening, and 100% of the resources are used for 1 to 1 minute; (2) when there are 99 people online, there is some transmission delay when the audio frequency is turned on, but the listening effect is good, and the resources of 1 to 2 minutes occupy 100%; (3) When there are 199 people online, there is a significant transmission delay when the audio is turned on, but it can still be listened to normally, and the resources occupy 100% in 2 to 4 minutes. Video performance test results: (1) when there are 19 people online, there is no delay in watching the video, and 100% of the resources are occupied for 1 to 2 minutes; (2) when there are 49 people online, there is some transmission delay when the video is opened, but the viewing effect is good, and the resources of 2 to 4 minutes occupy 100%; (3) when there are 99 people online, there is a significant transmission delay when it is turned on, but it can still be viewed normally, and the resources occupy 100% in 4 to 5 minutes.

### 4.3. Example Application and Analysis

This article organizes four sets of experiments to determine what wisdom users will produce when listening to songs. The first set of experiments initially established a list of adjectives describing the wisdom of music; the second set of experiments allowed the experimenters to vote on the wisdom words they felt, removing the wisdom words with a lower number of votes; the third and fourth groups tested the remaining wisdom words. The voting was conducted again to further reduce the number of wisdom words, and factor analysis was used to divide the remaining 33 wisdom words into 9 categories. In order to extract cepstrum parameters from music, the following steps are required: (1) Fourier transform the music signal to obtain the signal spectrum; (2) find the logarithm of the obtained spectrum; (3) then find the Fourier inverse transform, so that the cepstrum feature of music can be extracted. There are two main types of cepstrum features: (1) mel frequency cepstrum coefficient (MFCC); (2) perceptual linear prediction cepstrum extracted based on perceptual linear prediction (PLP) analysis. Studies have shown that these two cepstrum features can simulate the processing characteristics of the human ear to music signals. The spectrum centroid is a measure of the shape of the spectrum. It reflects the level of the audio frequency, and the two are in direct proportion. A large value of the spectrum centroid means a high frequency, and anyway, it is low. The audio frequency is closely related to wisdom. Usually, the spectrum centroid value of excited and passionate music is larger than that of peaceful and sad music.  Figure 7 shows a line chart comparing the centroid values of the music classroom test spectrum.

In order to test the capacity of the system for the number of candidates, 100-500 simultaneous online mock exams are arranged, mainly to test the performance of the system server for a large number of data processing requirements generated by a large number of candidates in the test process. After testing, it is found that the performance pressure of the test system occurs within 5-10 minutes of “starting the test” and “submitting the answer sheet.” Because there is minimal contact between the client and the server throughout the test, the server is under less stress. The following performance evaluation is made under the basic hardware environment and 100-question test environment, and the average value is calculated. The results of the experiment found that (1) only three examinations were conducted without examination papers and examination questions. The average pass rate of candidates was 85%, and the excellent rate (90 points and above) was 20%; (2) three examinations and the average pass rate of candidates for the analysis of test papers are 95%, and the excellent rate is 45%. (3) For students who have not conducted examination analysis, the average passing rate is 55% and the excellent rate is 5%; for students who have conducted examination analysis, the passing rate is 80% and the excellent rate is 30%.  Figure 8 shows the result of the failing rate in the music classroom test. It can be determined that the use of this system can greatly improve the quality of students' learning, is able to withstand the test of teaching practice, and is capable of assisting teaching tasks.

We store the state of the candidate in the state field of the student information table. If you have not taken the exam, the initial value is “0;” when the first login is successful, the value of this field is rewritten to “1,” which means that the answer is in the answer. The paper has not been handed in; if the paper has been turned in or the test time is up, the value of this field is changed to “2:” because it has been logged in, but the paper has not yet been handed in, the current value of this field is “l,” so it is when logging in for the second time, the invigilator must enter the password before continuing the exam. If you log in again after handing in the test paper, because the value of state is detected as “2,” it prompts “You have already handed in the paper, please do not log in again,” and then exit the program. After the computer is restarted, we log in to the examination system again, the original saved answers are not lost, so just open the question and continue to do the question. The test time is 100 minutes. The remaining time is saved in the test status table, and the remaining time is displayed on the screen. It is refreshed every 1 second. When it is a whole minute, the remaining minutes will be saved in the table once. When logging in again, we read the remaining time directly from the state table and display it on the answer window.

## 5. Conclusion

A multimodal smart music online teaching system and the implementation method for each module are introduced in this article. Uploading files in bulk requires a combination of multithreading, AJAX nonrefresh, and HTTP breakpoint resumable, as well as artificial intelligence to help extract information characteristics. Hierarchical relational databases are used in conjunction with object relationships to build the database structure, and multimedia data as well as simple binary data are used to complete the upload. To download and examine multimedia content while conserving resources, the point-to-point download concept is used with standard players. Experiments explore the relationship between audio and lyrics, while this paper's enhanced wireless network node feature selection technique and improved LFSM fusion method are both shown to be feasible and successful. The internal network environment has improved the security of the wireless network. Through the connection with the Internet and the integration of multimedia processing technology and storage technology, the limitation of the popularization and sharing of multimedia teaching resources in traditional management methods has been improved. To enable system migration and upgrading, a 4-tier structure is used in database design and system architecture. In addition, the system has also greatly improved the depth and breadth of data query. In this system, the application of BP neural wireless network technology can achieve good control of the huge test question database data in the system database, complex test attribute (chapter, difficulty, question type, knowledge points, etc.) association, etc., according to the teacher user's proposal. According to various requirements, the automatic or semiautomatic test paper composition function can be completed and the test results of students can be fed back and analyzed, which can efficiently and quickly improve the quality of students' learning and the teaching effect of teachers.

## Figures and Tables

**Figure 1:** Wireless network hierarchical topology.

**Figure 2:** Line graph of the efficiency of the online system decision tree.

**Figure 3:** Online teaching factor integration system.

**Figure 4:** Short-term average amplitude deviation statistics of music signals.

**Figure 5:** Fan-shaped distribution of the proportion of music periodic signals.

**Figure 6:** Occupancy rate curve of online teaching resources.

**Figure 7:** Line chart of the comparison of the centroid values of the spectrum of the music classroom test.

**Figure 8:** Result of failing rate in music classroom test.

**Table 1:** Interactive online teaching factors.

Factor index	Classification name	Test score	Weight
1	Instructional design	88	0.11
2	Teaching courseware	91	0.09
3	Expert comments	93	0.23
4	Teaching reflections	87	0.31
5	Student evaluations	94	0.26

## Data Availability

The data used to support the findings of this study are included within the article.
